The article "Evidence Summary of Temperature Management for Comatose Patients after Cardiopulmonary Resuscitation in ICUs" was retracted in 2023. Reasons: signs of a paper mill; compromised peer review; unreliable results or conclusions.

# Evidence Summary of Temperature Management for Comatose Patients after Cardiopulmonary Resuscitation in ICUs

**DOI:** 10.1155/2022/2220487

**Published:** 2022-06-30

**Authors:** Zhuo Yang, Ting Ni, Yan Yang, Hui Zhang, Hongli Chi

**Affiliations:** Department of EICU, The First Hospital of Jilin University, Changchun City, Jilin 130021, China

## Abstract

**Objective:**

This study aims to select and summarize the best evidence of temperature management for comatose patients after cardiopulmonary resuscitation in intensive care units (ICUs) at home and abroad.

**Method:**

Some well-known databases at home and abroad have been searched to find the guidelines, expert consensus, original documents, evidence summaries, and systematic evaluation about temperature management for comatose patients after cardiopulmonary resuscitation in ICUs. The databases included PubMed, Up to Date, Cochrane Library, the website of Registered Nurses' Association of Ontario, the Guideline Library of National Institute for Health and Clinical Excellence of the UK, China National Knowledge Infrastructure (CNKI), Wanfang Database, and VIP. The period for search is from the establishment of each database to the present. Two researchers who have received evidence-based nursing training and passed the examination evaluated, extracted, and integrated the literature quality with a blind method to summarize the best evidence.

**Results:**

A total of 10 pieces of literature were included in this study, including 4 in Chinese and 6 in English. Specifically, there were 4 guidelines, 1 expert consensus, 2 evidence summaries, 1 systematic evaluation, 1 literature review, and 1 comparative experiment, accounting for 40.0%, 10.0%, 20.0%, 10.0%, 10.0%, and 10.0%, respectively. The literature and materials were all qualified, and there was no heterogeneity and no significant publication bias in the included literature. The best evidence involved mild hypothermia therapy, rewarming, prevention of mild hypothermia-related complications, and nutritional support, with a total of 21 pieces of evidence (including 11, 3, 5, and 2 pieces of evidence, respectively). In terms of the recommendation grade, 7 pieces of evidence were at Grade A and 14 at Grade B.

**Conclusion:**

Health care providers should implement hypothermia management in comatose patients after cardiopulmonary resuscitation in ICUs, pay attention to the prevention of related complications, and provide enteral nutrition support.

## 1. Introduction

An intensive care unit (ICU) is a place for patients with severe illness or coma to receive diagnosis, treatment, and monitoring. It is also an important part of a medical organization. Cardiopulmonary resuscitation is a life-saving technique for patients with heart disease and respiratory arrest. It aims to restore patients' autonomous circulation and breathing and has been widely used in clinical practice [1]. The nursing after cardiopulmonary resuscitation in an ICU is of particular significance. It is necessary to restore patients' consciousness as soon as possible, stabilize circulation, promote the recovery of nutrition and metabolism, and maintain organs. For comatose patients receiving cardiopulmonary resuscitation in ICUs, scientific and comprehensive nursing can promote patients' recovery of consciousness, stabilize vital signs, and reduce mortality [2, 3]. Temperature management is an important nursing task for comatose patients after cardiopulmonary resuscitation in ICUs. Reasonable control of patients' temperature can reduce brain metabolism and inhibit immune-inflammatory response. At the same time, it features anticoagulation, inhibits apoptosis, reduces oxidative stress, and inhibits excitatory neurotoxicity [4, 5]. As a common temperature management strategy for critical patients in ICUs, mild hypothermia therapy has been widely recognized by scholars at home and abroad [6–8]. In view of this, this study summarizes the best evidence of the implementation of temperature management for comatose patients after cardiopulmonary resuscitation in ICUs at home and abroad to provide reference and guidance for the temperature management of such patients.

The article "Evidence Summary of Temperature Management for Comatose Patients after Cardiopulmonary Resuscitation in ICUs" was retracted in 2023. Reasons: signs of a paper mill; compromised peer review; unreliable results or conclusions.

## 2. Materials and Method

### 2.1. Issue Determination

Some well-known databases at home and abroad have been searched to find the guidelines, expert consensus, original documents, evidence summaries, and systematic evaluation about temperature management for comatose patients after cardiopulmonary resuscitation in ICUs. The search keywords included ICU, cardiopulmonary resuscitation, coma, and temperature management. Evidence-based theme: the effective temperature management for comatose patients after cardiopulmonary resuscitation in ICUs.

### 2.2. Literature Search

The up-down search was done according to the 6S Pyramid method. The databases included PubMed, Up to Date, Cochrane Library, the website of Registered Nurses' Association of Ontario, the Guideline Library of National Institute for Health and Clinical Excellence of the UK, China National Knowledge Infrastructure (CNKI), Wanfang Database, and VIP. The period for search was from the establishment of each database to the present.

### 2.3. Inclusion and Exclusion Criteria for Literature

Inclusion criteria: ①the subjects were comatose patients admitted to the ICU after cardiac arrest cardiopulmonary resuscitation; ②the subjects were all adult patients aged 18 to 60 years; ③ the literature involved temperature management; ④the types of literature included guidelines, expert consensus, original document, evidence summary, and systematic evaluation; ⑤ the literature is in Chinese or English.

The article "Evidence Summary of Temperature Management for Comatose Patients after Cardiopulmonary Resuscitation in ICUs" was retracted in 2023. Reasons: signs of a paper mill; compromised peer review; unreliable results or conclusions.

Exclusion criteria: ① the type of literature was draft or abstract only; ② the subjects had certain diseases such as thermoregulatory disorder; ③literature information was incomplete; ④literature failed to meet the evaluation criteria of Joanna Briggs Institute (JBI) in terms of quality.

### 2.4. Literature Quality Evaluation

Two researchers who have received evidence-based nursing training and passed the examination evaluated, extracted, and integrated the literature quality with a blind method. If they had the same judgment, the decision would be final. If not, arbitration was made by the evidence-based care team in the hospital. The principle of literature quality evaluation was: preference was given to high-quality evidence, the latest evidence published in authoritative journals, and evidence-based evidence. AMSTAR 2.0 was used to evaluate the included literature on expert consensus, evidence summary, and systematic evaluation. The evaluation method includes 16 entries, of which 7 key entries (entries 2/4/7/9/11/13/15): literature with no or only 1 nonkey entry nonconformity is considered high quality; literature with more than 1 nonkey entry nonconformity is considered medium quality; literature with 1 or more key entries nonconformity with or without nonkey entry nonconformity is considered low quality. High-quality and moderate-quality documents are considered to be up to standard.

The included guidelines were evaluated by AGREE II, and the included literature review, comparative experiment, and original literature were evaluated by RevMan 5.3.

### 2.5. Statistical Methods

Heterogeneity tests and risk of bias analyses were performed using RevMan 5.3 software. The included literature was considered not significantly heterogeneous if the Q Statistic *P* > 0.1. The percentage of heterogeneity in the overall study was expressed as *I*^2^, and the effect size was expressed as 95% confidence interval (CI). *P* < 0.05 was considered a statistically significant difference.

## 3. Results

### 3.1. General Description of the Included Literature

A total of 77 literatures were retrieved. Eighteen studies with cases and abstracts only were removed, four articles with subjects with thermoregulatory disorders were excluded, and 26 articles with incomplete information and 19 articles that did not meet the JBI evaluation criteria were removed. Finally, 10 studies were included [9–18]. The flow chart of literature inclusion is shown in Figure 1. Four of the 10 studies were in Chinese and six were in English. Specifically, there were 4 guidelines, 1 expert consensus, 2 evidence summaries, 1 systematic evaluation, 1 literature review, and 1 comparative experiment, accounting for 40.0%, 10.0%, 20.0%, 10.0%, 10.0%, and 10.0%, respectively. All the literature and materials were qualified. See Table 1 for details.

The article "Evidence Summary of Temperature Management for Comatose Patients after Cardiopulmonary Resuscitation in ICUs" was retracted in 2023. Reasons: signs of a paper mill; compromised peer review; unreliable results or conclusions.

In addition, after statistical analysis, there was no heterogeneity in the included literature (*I*^2^ = 0.24, *P* = 0.77) and no significant publication bias, as shown in Figure 2.

### 3.2. Best Evidence Summary of Temperature Management for Comatose Patients after Cardiopulmonary Resuscitation in ICUs

The best evidence involved mild hypothermia therapy, rewarming, prevention of mild hypothermia-related complications, and nutritional support, with a total of 21 pieces of evidence (including 11, 3, 5, and 2 pieces of evidence, respectively). In terms of the recommendation grade, 7 pieces of evidence were at Grade A and 14 at Grade B. See Table 2 for details.

## 4. Discussion

### 4.1. Significance of Evidence Summary of Temperature Management for Comatose Patients after Cardiopulmonary Resuscitation in ICUs

As an important nursing operation for comatose patients after cardiopulmonary resuscitation in ICUs, temperature management is of positive significance in promoting the prognosis and improving the prognosis [19]. Hypothermia therapy has become a recognized intervention measure for critical patients in ICUs, and there is a lot of supporting evidence at home and abroad. However, there is still a lack of the best evidence for the temperature management of comatose patients after cardiopulmonary resuscitation in ICUs. The implementation of this operation helps guide the nursing and makes the operation more standardized and reasonable, ensuring real temperature management.

### 4.2. Analysis of Evidence Summary of Temperature Management for Comatose Patients after Cardiopulmonary Resuscitation in the ICU

A total of 10 pieces of evidence on temperature management of comatose patients after cardiopulmonary resuscitation in ICUs were included in this study. The literature was qualified, ensuring the preciseness and repeatability of the results of the study. Based on the evidence summary of the included literature, it was found that the temperature management of comatose patients after cardiopulmonary resuscitation in ICUs involved mild hypothermia therapy, rewarming, prevention of mild hypothermia-related complications, and nutritional support. Specifically, 11 pieces of evidence were related to mild hypothermia therapy (recommendation grade: 6 pieces at Grade A and 5 pieces at Grade B); 3 pieces of evidence were related to rewarming (recommendation grade: Grade B); 5 pieces of evidence were related to the prevention of mild hypothermia-related complications (recommendation grade: Grade B); and 2 pieces of evidence were related to nutritional support (recommendation grade: 1 piece at Grade A and 1 piece at Grade B). In addition, the results of the best evidence summary of this study included the indications, contraindications, place of implementation, implementation personnel, start time, target temperature, cooling measures, duration of induced hypothermia, body temperature monitoring methods, and interruption of mild hypothermia therapy, helping nursing personnel screen the target population requiring mild hypothermia therapy and defining the implementation standard of this therapy from all aspects as the core content to guide its popularization and application in clinical practice. In terms of rewarming, the requirements for rewarming speed, body temperature after rewarming, and duration of maintenance clarified the precautions for rewarming after mild hypothermia therapy, ensuring that the patients' body temperature returned to normal in a slow and stable manner and guaranteeing the recovery of physiological and metabolic state. The prevention of mild hypothermia-related complications included the evaluation and control of shivering, the monitoring and treatment of arrhythmia, the monitoring and control of infection, and the monitoring of serum potassium level and the prevention of other complications. It could provide guidance to the medical staff in monitoring the vital signs of patients, ensuring that the patients safely receive mild hypothermia therapy and avoiding any secondary injury caused by complications. Nutritional support included guidance on enteral nutrition and energy intake, ensuring the nutritional supply of patients and avoiding various problems caused by insufficient or excess nutrition. In consideration of previous studies and the author's working experience, it is recommended to strictly refer to the above items and evidence to support the implementation of temperature management for comatose patients after cardiopulmonary resuscitation in ICUs. A study [20] confirmed that mild hypothermia therapy could improve the success rate of cardiopulmonary resuscitation in ICUs, provide brain protection, and improve brain metabolism and microcirculation. Another report [21] showed that, compared with conventional temperature management, mild hypothermia therapy could promote the rapid recovery of comatose patients after cardiopulmonary resuscitation and reduce the neurological deficit.

The article "Evidence Summary of Temperature Management for Comatose Patients after Cardiopulmonary Resuscitation in ICUs" was retracted in 2023. Reasons: signs of a paper mill; compromised peer review; unreliable results or conclusions.

However, there are still some limitations in this study: (i) there is still room for optimization of the temperature management scheme for comatose patients after cardiopulmonary resuscitation in the ICU, and how to further optimize it to speed up recovery remains to be explored; (ii) patients of different age groups may have different needs for temperature management, and the follow-up study still needs to be refined.

## 5. Conclusion

For comatose patients after cardiopulmonary resuscitation in ICUs, it is recommended that the indications, contraindications, place of implementation, implementation personnel, start time, target temperature, cooling measures, duration of induced hypothermia, body temperature monitoring methods, interruption of mild hypothermia therapy, rewarming speed, requirements for body temperature and duration of maintenance after rewarming, evaluation and control of shivering, monitoring and treatment of arrhythmia, monitoring and control of infection, monitoring of serum potassium level and prevention of other complications, nutritional support, and other relevant evidence should be referred to in order to support the implementation of body temperature management, so as to promote the prognosis of patients.

## Figures and Tables

**Figure 1:** Flow chart of literature inclusion.

**Figure 2:** Funnel plot for analysis of publication bias in the included literature.

**Table 1:** General description of the included literature.

Author	Year of publication	Title	Type	Source	Language	Quality evaluation
Hu Chunlin, et al. [9]	2009	Meta-analysis of mild hypothermia therapy in cardiopulmonary resuscitation after cardiac arrest	Systematic evaluation	Wanfang Database	Chinese	Qualified
Yu Tao et al. [10]	2011	Advances in hypothermia therapy during cardiopulmonary resuscitation	Literature review	CNKI	Chinese	Qualified
American Heart Association [11]	2015	Web-based integrated guidelines for cardiopulmonary resuscitation and emergency cardiovascular care– part 8:post-cardiac arrest care	Guideline	PubMed	English	Qualified
Nolan et al. [12]	2015	European Resuscitation Council and European Society of Intensive Care Medicine guidelines for post-resuscitation care 2015:section 5 of the European Resuscitation Council Guidelines for Resuscitation 2015	Guideline	PubMed	English	Qualified
ARC [13]	2016	ANZCOR Guideline 1 1.8 – targeted temperature management (TTM) after cardiac arrest	Guideline	Cochrane Library	English	Qualified
Howes et al. [14]	2016	Canadian Guidelines for the use of targeted temperature management (therapeutic hypothermia) after cardiac arrest: a joint statement from The Canadian Critical Care Society (CCCS), Canadian Neurocritical Care Society (CNCCS), and the Canadian Critical Care Trials Group (CCCTG)	Comparative experiment	The website of Registered Nurses' Association of Ontario	English	Qualified
Geocadin et al. [15]	2017	Practice guideline summary: reducing brain injury following cardiopulmonary resuscitation: report of the Guideline Development, Dissemination, and Implementation Subcommittee of the American Academy of Neurology	Guideline	PubMed	English	Qualified
Cariou et al. [16]	2017	Targeted temperature management in the ICU: guidelines from a French expert panel	Expert consensus	Up to Date	English	Qualified
Zhang Yuman et al. [17]	2020	Summary of the best evidence of target body temperature management for patients with cardiac arrest	Evidence summary	Wanfang Database	Chinese	Qualified
Song Chunxia et al. [18]	2021	Quality evaluation of target body temperature management guidelines for patients with cardiac arrest	Evidence summary	VIP	Chinese	Qualified

The article "Evidence Summary of Temperature Management for Comatose Patients after Cardiopulmonary Resuscitation in ICUs" was retracted in 2023. Reasons: signs of a paper mill; compromised peer review; unreliable results or conclusions.

**Table 2:** Best evidence summary of temperature management for comatose patients after cardiopulmonary resuscitation in ICUs.

Item	Evidence	Recommendation grade
Mild hypothermia therapy	Indications: Mild hypothermia therapy should be implemented as soon as possible for adult patients who recover spontaneous circulation but are still in a coma after cardiac arrest.	Grade A
	Contraindications: No absolute contraindications. The relative contraindications include severe infection, uncontrollable bleeding, and intractable shock.	Grade A
	Place of implementation: With necessary support, it can be initiated in pre-hospital settings, emergencyrooms, and ICUs.	Grade A
	Implementation personnel: It is recommended that the on-site medical staff who have received the training on mild hypothermia therapy start the treatment as soon as possible without the specialist consultation.	Grade A
	Start time: It should be initiated within 6 hours after the recovery of autonomic circulation, and the earlier, the better. If inevitable delay occurs due to various reasons, it may still be beneficial within 8 or more hours after the recovery of autonomic circulation.	Grade A
	Target temperature: 33°C (32°C-34°C) is recommended for patients in a deep coma, or with evidence of brain edema or malignant EEG waveform. Otherwise, the recommended temperature is <36°C (32°C-36°C).	Grade B
	Cooling measures: The whole-body hypothermia technique with temperature feedback control device or intravascular hypothermia technique or locally induced hypothermia (head) which gradually spreads to the whole body. If the medical conditions are undesirable, ice blanket, ice cap, and other treatments can be used. In case of cardiac insufficiency or risk of pulmonary edema, be careful to use 4°C normal saline intravenous infusion for induction.	Grade B
	Duration of induced hypothermia: The target temperature shall be reached as soon as possible, and the recommended duration is 2-4 hours.	Grade B
	Duration of hypothermia maintenance: 24 hours are recommended.	Grade B
	Temperature monitoring method: Bladder or rectum temperature monitoring is the first choice, and nasopharynx, esophagus, bladder, endotracheal tube cuff, and pulmonary artery are recommended as the core monitoring sites.	Grade A
	Interruption of mild hypothermia therapy: It is recommended to interrupt mild hypothermia therapy for patients with unstable hemodynamics, ineffective active resuscitation, and severe bleeding during treatment	Grade B
Rewarming	Rewarming speed: 0.25°C-0.5 °C/h is recommended	Grade B
	Temperature requirement after rewarming: <37.5 °C	Grade B
	Duration of maintenance after rewarming: Rewarming shall be maintained until 72 hours after resuscitation	Grade B
Prevention of mild hypothermia-related complications	Evaluation and control of shivering: Bedside shivering assessment scale (BSAS) and continuous EEG monitoring assessment are selected. It is recommended to administrate muscle relaxant buspirone (load: 30 mg; maintenance dose: 15 mg, once every 8 h), midazolam (load: 0.1 mg/kg; maintenance dose: 2-6 mg/h) and pethidine hydrochloride (load: 1 mg/kg; maintenance dose: 25-45 mg/h) alone or in combination. If shivering is not controlled as expected or rapid cooling occurs, vecuronium bromide (load: 0.03-0.05 mg/kg; maintenance dose: 0.02-0.03 mg/kg·h) or rocuronium bromide (load 0.6 mg/kg, maintenance dose 0.3-0.6 mg/kg·h) should be added. It is not recommended to routinely use anticonvulsant drugs to prevent epilepsy. At the same time, active body surface warming should be made and sedation and analgesia should be provided.	Grade B
	Monitoring and treatment of arrhythmia: Monitor ECG, carefully use drugs that can prolong QTc interval, and use antiarrhythmic drugs for arrhythmias that are malignant or seriously affect hemodynamics. If bradycardia occurs, routine treatment is not recommended unless it leads to hemodynamic instability.	Grade B
	Monitoring and control of infection: It is not allowed to use procalcitonin to diagnose infection during mild hypothermia therapy, and antibiotics are also prohibited. It is recommended to operate in strict accordance with disinfection procedures.	Grade B
	Monitoring of serum potassium level: The recommended serum potassium level is >3.0 mmol/L.	Grade B
	Prevention of other complications: Low metabolic rate, abnormal blood glucose, cold diuresis, hemodynamic instability, coagulation disorder, and decreased drug clearance may occur. Therefore, the patients should be closely monitored and actively treated.	Grade B
Nutritional support	Enteral nutrition: Enteral nutrition support is recommended during mild hypothermia therapy.	Grade A
	Energy intake: It is recommended to keep the energy intake up to 75% of the target value under normal body temperature during mild hypothermia therapy.	Grade B

Note: Grade A indicates strong recommendation; Grade B indicates recommendation.

The article "Evidence Summary of Temperature Management for Comatose Patients after Cardiopulmonary Resuscitation in ICUs" was retracted in 2023. Reasons: signs of a paper mill; compromised peer review; unreliable results or conclusions.

## Data Availability

The data used to support the findings of this study are available from the corresponding author upon request.
